# Comparison of Five Methods to Estimate the Parameters for the Three-Parameter Lindley Distribution with Application to Life Data

**DOI:** 10.1155/2021/2689000

**Published:** 2021-12-08

**Authors:** Mathil K. Thamer, Raoudha Zine

**Affiliations:** ^1^Laboratory of Probability and Statistics, Faculty of Sciences of Sfax, Sfax, Tunisia; ^2^Department of Economics, College of Administration and Economics, University of Anbar, Iraq

## Abstract

We have studied one of the most common distributions, namely, Lindley distribution, which is an important continuous mixed distribution with great ability to represent different systems. We studied this distribution with three parameters because of its high flexibility in modelling life data. The parameters were estimated by five different methods, namely, maximum likelihood estimation, ordinary least squares, weighted least squares, maximum product of spacing, and Cramér-von Mises. Simulation experiments were performed with different sample sizes and different parameter values. The different methods were compared on the generated data by mean square error and mean absolute error. In addition, we compared the methods for real data, which represent COVID-19 data in Iraq/Anbar Province.

## 1. Introduction

The Lindley distribution was proposed in 1958 by Lindley [1]; however, actual interest began in 2008 when Ghitany et al. [2] studied its properties and applications. Since then, this distribution has been developed as generalised Lindley distribution in 2009 by Zakerzadeh & Dolati [3], a two-parameter Lindley distribution in 2013 by Shanker et al. [4], another two-parameter Lindley distribution in the same year by Shanker & Mishra [5], Lindley distribution with a location parameter as a three-parameter distribution in 2016 by Abd El-Monsef [6], and another three-parameter Lindley distribution in 2017 by Shanker et al. [4].

The Lindley distribution is made up of mixing two continuous distributions with different weights; the first is exponential distribution with *θ*, and the second is gamma distribution with 2 and *θ*, that is,

(1) $$\begin{array}{c} f\left(x;\theta \right)=wf_{1}\left(x;\theta \right)+\left(1-w\right)f_{2}\left(x;\theta \right), \end{array}$$

where

(2) $$\begin{array}{c} f_{1}\left(x;\theta \right)=\theta e^{-\theta x},\\ f_{2}\left(x;\theta \right)=\theta^{2}xe^{-\theta x}. \end{array}$$

Thus, the resulting function is as follows:

(3) $$\begin{array}{c} f\left(x;\theta \right)=w\theta e^{-\theta x}+\left(1-w\right)\theta^{2}xe^{-\theta x}. \end{array}$$

Lindley [1] used *w* = *θ*/(*θ* + 1); hence, the probability density function (p.d.f.) is as follows:

(4) $$\begin{array}{c} f\left(x;\theta \right)=\frac{\theta^{2}}{\theta +1}\left(1+x\right)e^{-\theta x},\;x>0,\theta \geq 0. \end{array}$$

Ghitany et al. [2] introduced its cumulative distribution function (c.d.f.) as follows:

(5) $$\begin{array}{c} F\left(x;\theta \right)=1-\left[\frac{\theta +1+\theta x}{\theta +1}\right]e^{-\theta x}. \end{array}$$

Parameter estimation of the two-parameter Lindley distribution was conducted by many researchers, such as Al-Bayati [7], Sharafi [8], and Demirci Biçer [9]. However, the parameters of the three-parameter Lindley distribution were only estimated in the maximum likelihood method be Shanker et al. [10]. Therefore, in this research, the distribution parameters were estimated using different methods.

## 2. Materials and Methods

### 2.1. The Three-Parameter Lindley Distribution

The three-parameter Lindley distribution (THPL) was proposed by Shanker et al. [10]; the weight *w* = *αθ*/(*αθ* + *β*) was used, as follows:

(6) $$\begin{array}{c} f\left(x;\alpha ,\beta ,\theta \right)=\frac{\alpha \theta }{\alpha \theta +\beta }\theta e^{-\theta x}+\frac{\beta }{\alpha \theta +\beta }\theta^{2}xe^{-\theta x}, \end{array}$$

resulting in the following:

(7) $$\begin{array}{c} f\left(x;\theta ,\alpha ,\beta \right)=\frac{\theta^{2}}{\alpha \theta +\beta }\left(\alpha +\beta x\right)e^{-\theta x},\;x,\theta ,\beta >0\text{ and }\alpha \theta +\beta >0, \end{array}$$

(8) $$\begin{array}{c} F\left(x;\theta ,\alpha ,\theta \right)=1-\left[\frac{\alpha \theta +\beta +\beta \theta x}{\alpha \theta +\beta }\right]e^{-\theta x},\;x,\theta ,\beta >0\text{ and }\alpha \theta +\beta >0. \end{array}$$

Figures 1 and 2 show the p.d.f. and c.d.f. for different parameter values.

The quantile function of the three-parameter Lindley distribution is given by the following:

(9) $$\begin{array}{c} F\left(x;\theta ,\alpha ,\beta \right)=1-\left[\frac{\alpha \theta +\beta +\beta \theta x}{\alpha \theta +\beta }\right]e^{-\theta x}=u\Rightarrow 1-u=\left[\frac{\alpha \theta +\beta +\beta \theta x}{\alpha \theta +\beta }\right]e^{-\theta x}\Rightarrow \left(\alpha \theta +\beta \right)\left(1-u\right)=\left[\alpha \theta +\beta +\beta \theta x\right]e^{-\theta x}\Rightarrow \frac{\left(\alpha \theta +\beta \right)\left(1-u\right)}{\beta }=\left[\frac{\alpha \theta +\beta }{\beta }+\theta x\right]e^{-\theta x}\Rightarrow -\frac{\left(\alpha \theta +\beta \right)\left(1-u\right)e^{-\left(\left(\alpha \theta +\beta \right)/\beta \right)}}{\beta }=-\left[\frac{\alpha \theta +\beta }{\beta }+\theta x\right]e^{-\left(\theta x+\left(\left(\alpha \theta +\beta \right)/\beta \right)\right)}\Rightarrow W_{-1}\left[-\frac{\left(\alpha \theta +\beta \right)\left(1-u\right)e^{-\left(\left(\alpha \theta +\beta \right)/\beta \right)}}{\beta }\right]=-\left[\frac{\alpha \theta +\beta }{\beta }+\theta x\right], \end{array}$$

(10) $$\begin{array}{c} ∴x=Q\left(u;\theta ,\alpha ,\beta \right)=-\frac{\alpha }{\beta }-\frac{1}{\theta }-\frac{1}{\theta }W_{-1}\left[-\frac{\left(\alpha \theta +\beta \right)\left(1-u\right)e^{-\left(\left(\alpha \theta +\beta \right)/\beta \right)}}{\beta }\right],\;0<u<1, \end{array}$$

where *W*_−1_(.) denotes the negative branch of the Lambert *W* function.

### 2.2. Several Estimators of the Parameters of THPL Distribution

We present five well-known methods to estimate the parameters of the three-parameter Lindley distribution, including maximum-likelihood (ML), ordinary least-squares (OLS), weighted least-squares (WLS), maximum product of spacing (MPS), and Cramér-von Mises (CVM).

### 2.3. Maximum Likelihood Estimators

The log-likelihood of the positive vector of observations *x* = (*x*_1_, *x*_2_, ⋯, *x*_*n*_) under the three-parameter Lindley distribution can be written as follows:

(11) $$\begin{array}{c} \ell \left(\theta ,\alpha ,\beta \right)=2nln\theta -nln\left(\alpha \theta +\beta \right)+\overset{n}{\underset{i=1}{\sum }}\ln\left(\alpha +\beta x_{i}\right)-n\theta \overset{¯}{x}, \end{array}$$

where $\overset{¯}{x}$ is the sample mean.

Shanker et al. [10] derived the maximum likelihood estimates (MLE) $\hat{\theta },\hat{\alpha },$ and $\hat{\beta }$ of *θ*, *α*, and *β*, by solving the following nonlinear equations:

(12) $$\begin{array}{c} \frac{\partial \ell \left(\theta ,\alpha ,\beta \right)}{\partial \theta }=\frac{2n}{\theta }-\frac{n\alpha }{\alpha \theta +\beta }-n\overset{¯}{x}=0,\\ \frac{\partial \ell \left(\theta ,\alpha ,\beta \right)}{\partial \alpha }=\frac{-n\theta }{\alpha \theta +\beta }+\overset{n}{\underset{i=1}{\sum }}\frac{1}{\alpha +\beta x_{i}}=0,\\ \frac{\partial \ell \left(\theta ,\alpha ,\beta \right)}{\partial \beta }=\frac{-n}{\alpha \theta +\beta }+\overset{n}{\underset{i=1}{\sum }}\frac{x_{i}}{\alpha +\beta x_{i}}=0. \end{array}$$

We can also obtain MLE by maximising (11) via fminunc function in MATLAB.

### 2.4. Ordinary and Weighted Least-Square Estimators

Suppose that *X*_(1)_ ≤ *X*_(2)_ ≤ ⋯≤*X*_(*n*)_ are the order statistics of a random sample from any probability distribution. The *i*^th^-order statistic has the mean and the variance as follows:

(13) $$\begin{array}{c} E\left[F\left(X_{\left(i\right)}\right)\right]=\frac{i}{n+1}\text{ and }\mathrm{var}\left[F\left(X_{\left(i\right)}\right)\right]=\frac{i\left(n-i+1\right)}{{\left(n+1\right)}^{2}\left(n+2\right)},\;\forall i\in 1,2,\cdots ,n. \end{array}$$

OLS and WLS were proposed in 1988 by Swain et al. [11]. We can get OLS estimates for the parameters by minimising the following function with respect to the parameters, as follows:

(14) $$\begin{array}{c} R=\overset{n}{\underset{i=1}{\sum }}{\left[F\left(x_{\left(i\right)}\right)-F\left(i\right)\right]}^{2}, \end{array}$$

where *F*(*x*_(*i*)_) represents the theoretical c.d.f. of the observation *x*_(*i*)_ of the distribution under study and *ℱ*(*i*) represents the empirical c.d.f. which is usually estimated by $\hat{ℱ}\left(i\right)=i/\left(n+1\right)$; then, we obtain the following:

(15) $$\begin{array}{c} R=\overset{n}{\underset{i=1}{\sum }}{\left[F\left(x_{\left(i\right)}\right)-\frac{i}{n+1}\right]}^{2}. \end{array}$$

This function can be obtained for the three-parameter Lindley distribution after substituting for *F*(*x*_(*i*)_) in the previous equation by its c.d.f. defined in equation (8), as follows:

(16) $$\begin{array}{c} R\left(\theta ,\alpha ,\beta \right)=\overset{n}{\underset{i=1}{\sum }}{\left[\left(\frac{\alpha \theta +\beta +\beta \theta x_{\left(i\right)}}{\alpha \theta +\beta }\right)e^{-\theta x_{\left(i\right)}}-\frac{n+1-i}{n+1}\right]}^{2}. \end{array}$$

We can determine the OLS estimates by minimising (16) with respect to the parameters via fminunc function or by solving the following equations:

(17) $$\begin{array}{c} \frac{\partial R\left(\theta ,\alpha ,\beta \right)}{\partial \theta }=\overset{n}{\underset{i=1}{\sum }}\left[\left(\frac{\alpha \theta +\beta +\beta \theta x_{\left(i\right)}}{\alpha \theta +\beta }\right)e^{-\theta x_{\left(i\right)}}-\frac{n+1-i}{n+1}\right]\left[\theta \alpha^{2}x_{\left(i\right)}\theta \alpha \beta x_{\left(i\right)}^{2}+2\alpha \beta x_{\left(i\right)}^{2}+\beta^{2}x_{\left(i\right)}\right]e^{-\theta x_{\left(i\right)}}=0,\\ \frac{\partial S\left(\theta ,\alpha ,\beta \right)}{\partial \alpha }=\overset{n}{\underset{i=1}{\sum }}\left[\left(\frac{\alpha \theta +\beta +\beta \theta x_{\left(i\right)}}{\alpha \theta +\beta }\right)e^{-\theta x_{\left(i\right)}}-\frac{n+1-i}{n+1}\right]x_{\left(i\right)}e^{-\theta x_{\left(i\right)}}=0,\\ \frac{\partial S\left(\theta ,\alpha ,\beta \right)}{\partial \beta }=\overset{n}{\underset{i=1}{\sum }}\left[\left(\frac{\alpha \theta +\beta +\beta \theta x_{\left(i\right)}}{\alpha \theta +\beta }\right)e^{-\theta x_{\left(i\right)}}-\frac{n+1-i}{n+1}\right]x_{\left(i\right)}e^{-\theta x_{\left(i\right)}}=0. \end{array}$$

We can obtain WLS estimates for the parameters by minimising the following function with respect to the parameters:

(18) $$\begin{array}{c} W=\overset{n}{\underset{i=1}{\sum }}w_{i}{\left[F\left(x_{\left(i\right)}\right)-F\left(i\right)\right]}^{2},\;w_{i}=\frac{{\left(n+1\right)}^{2}\left(n+2\right)}{i\left(n+1-i\right)}. \end{array}$$

This function can be obtained for the three-parameter Lindley distribution after substituting for *F*(*x*_(*i*)_) in the previous equation by its c.d.f. defined in equation (8), as follows:

(19) $$\begin{array}{c} W\left(\theta ,\alpha ,\beta \right)={\left(n+1\right)}^{2}\left(n+2\right)\overset{n}{\underset{i=1}{\sum }}\frac{{\left[\left(\left(\alpha \theta +\beta +\beta \theta x_{\left(i\right)}\right)/\left(\alpha \theta +\beta \right)\right)e^{-\theta x_{\left(i\right)}}-\left(\left(n+1-i\right)/\left(n+1\right)\right)\right]}^{2}}{i\left(n+1-i\right)}. \end{array}$$

WLS estimates can be obtained by minimising (19) with respect to the parameters via fminunc function or by solving the following equations:

(20) $$\begin{array}{c} \frac{\partial W\left(\theta ,\alpha ,\beta \right)}{\partial \theta }=\overset{n}{\underset{i=1}{\sum }}\left[\left(\frac{\alpha \theta +\beta +\beta \theta x_{\left(i\right)}}{\alpha \theta +\beta }\right)e^{-\theta x_{\left(i\right)}}-\frac{n+1-i}{n+1}\right]\frac{\left[\theta \alpha^{2}x_{\left(i\right)}+\theta \alpha \beta x_{\left(i\right)}^{2}+2\alpha \beta x_{\left(i\right)}^{2}+\beta^{2}x_{\left(i\right)}\right]e^{-\theta x_{\left(i\right)}}}{i\left(n+1-i\right)}=0,\\ \frac{\partial W\left(\theta ,\alpha ,\beta \right)}{\partial \alpha }=\overset{n}{\underset{i=1}{\sum }}\left[\left(\frac{\alpha \theta +\beta +\beta \theta x_{\left(i\right)}}{\alpha \theta +\beta }\right)e^{-\theta x_{\left(i\right)}}-\frac{n+1-i}{n+1}\right]\frac{x_{\left(i\right)}e^{-\theta x_{\left(i\right)}}}{i\left(n+1-i\right)}=0,\\ \frac{\partial W\left(\theta ,\alpha ,\beta \right)}{\partial \beta }=\overset{n}{\underset{i=1}{\sum }}\left[\left(\frac{\alpha \theta +\beta +\beta \theta x_{\left(i\right)}}{\alpha \hat{\theta }+\hat{\beta }}\right)e^{-\theta x_{\left(i\right)}}-\frac{n+1-i}{n+1}\right]\frac{x_{\left(i\right)}e^{-\theta x_{\left(i\right)}}}{i\left(n+1-i\right)}=0. \end{array}$$

### 2.5. Maximum Product of Spacing Estimators

MPS was derived by Cheng & Amin in 1979 [12]; the idea of this method is to maximise the following function:

(21) $$\begin{array}{c} P=\frac{1}{n+1}\overset{n+1}{\underset{i=1}{\sum }}\log D_{i}, \end{array}$$

where *D*_*i*_ = *F*(*x*_(*i*)_) − *F*(*x*_(*i* − 1)_) and *F*(*x*_(0)_) = 0; *F*(*x*_(*n* + 1)_) = 1.

This function can be obtained for the three-parameter Lindley distribution after substituting for *F*(*x*_(*i*)_) in the previous equation by its c.d.f. defined in equation (8), as follows:

(22) $$\begin{array}{c} P\left(\theta ,\alpha ,\beta \right)=\frac{1}{n+1}\overset{n+1}{\underset{i=1}{\sum }}\log\left[Q_{i}\right]-\log\left(\alpha \theta +\beta \right), \end{array}$$

where

(23) $$\begin{array}{c} Q_{i}=\alpha \theta \left[e^{-\theta x_{\left(i-1\right)}}-e^{-\theta x_{\left(i\right)}}\right]+\beta \left[e^{-\theta x_{\left(i-1\right)}}-e^{-\theta x_{\left(i\right)}}\right]+\beta \theta \left[x_{\left(i-1\right)}e^{-\theta x_{\left(i-1\right)}}-x_{\left(i\right)}e^{-\theta x_{\left(i\right)}}\right]. \end{array}$$

We can identify the MPS estimates by maximising (22) via fminunc function or by solving the following equations:

(24) $$\begin{array}{c} \frac{\partial P\left(\theta ,\alpha ,\beta \right)}{\partial \theta }=\frac{1}{n+1}\overset{n}{\underset{i=1}{\sum }}\frac{1}{Q_{i}}\frac{\partial Q_{i}}{\partial \theta }-\frac{\alpha }{\alpha \theta +\beta }=0,\\ \frac{\partial P\left(\theta ,\alpha ,\beta \right)}{\partial \alpha }=\frac{1}{n+1}\overset{n}{\underset{i=1}{\sum }}\frac{1}{Q_{i}}\frac{\partial Q_{i}}{\partial \alpha }-\frac{\theta }{\alpha \theta +\beta }=0,\\ \frac{\partial P\left(\theta ,\alpha ,\beta \right)}{\partial \beta }=\frac{1}{n+1}\overset{n}{\underset{i=1}{\sum }}\frac{1}{Q_{i}}\frac{\partial Q_{i}}{\partial \beta }-\frac{1}{\alpha \theta +\beta }=0, \end{array}$$

where

(25) $$\begin{array}{c} \frac{\partial Q_{i}}{\partial \theta }=\alpha \left[\left(e^{-\theta x_{\left(i-1\right)}}-e^{-\theta x_{\left(i\right)}}\right)-\theta \left(x_{\left(i-1\right)}e^{-\theta x_{\left(i-1\right)}}-x_{\left(i\right)}e^{-\theta x_{\left(i\right)}}\right)\right]+\beta \left[\left(x_{\left(i-1\right)}e^{-\theta x_{\left(i-1\right)}}-x_{\left(i\right)}e^{-\theta x_{\left(i\right)}}\right)-\theta \left(x_{\left(i-1\right)}^{2}e^{-\theta x_{\left(i-1\right)}}-x_{\left(i\right)}^{2}e^{-\theta x_{\left(i\right)}}\right)\right],\\ \frac{\partial Q_{i}}{\partial \alpha }=\theta \left(e^{-\theta x_{\left(i-1\right)}}-e^{-\theta x_{\left(i\right)}}\right),\\ \frac{\partial Q_{i}}{\partial \beta }=\left(e^{-\theta x_{\left(i-1\right)}}-e^{-\theta x_{\left(i\right)}}\right)+\theta \left(x_{\left(i-1\right)}e^{-\theta x_{\left(i-1\right)}}-x_{\left(i\right)}e^{-\theta x_{\left(i\right)}}\right). \end{array}$$

Note that if there is a tie, we cannot find the natural logarithm of *D*_*i*_ for the corresponding observation. Thus, we replace *D*_*i*_with the observation's p.d.f., that is, *D*_*i*_ = *f*(*x*_(*i*)_).

### 2.6. Cramér-von Mises Estimators

CVM was proposed by MacDonald in 1971 [13]. The idea of this method is to minimise the following function:

(26) $$\begin{array}{c} C=\frac{1}{12n}+\overset{n}{\underset{i=1}{\sum }}{\left[F\left(x_{\left(i\right)}\right)-\frac{2i-1}{2n}\right]}^{2}. \end{array}$$

This function can be obtained for the three-parameter Lindley distribution after substituting for *F*(*x*_(*i*)_) in the previous equation by its c.d.f., which was defined in equation (8), as follows:

(27) $$\begin{array}{c} C\left(\theta ,\alpha ,\beta \right)=\frac{1}{12n}+\overset{n}{\underset{i=1}{\sum }}{\left[\left(\frac{\alpha \theta +\beta +\beta \theta x_{\left(i\right)}}{\alpha \theta +\beta }\right)e^{-\theta x_{\left(i\right)}}-\frac{2n+1-2i}{2n}\right]}^{2}. \end{array}$$

We can determine the CVM estimates by maximising (27) via fminunc function or by solving the following equations:

(28) $$\begin{array}{c} \frac{\partial C\left(\theta ,\alpha ,\beta \right)}{\partial \theta }=\overset{n}{\underset{i=1}{\sum }}\left[\left(\frac{\alpha \theta +\beta +\beta \theta x_{\left(i\right)}}{\alpha \hat{\theta }+\beta }\right)e^{-\theta x_{\left(i\right)}}-\frac{2n+1-2i}{2n}\right]\left[\theta \alpha^{2}x_{\left(i\right)}+\theta \alpha \beta x_{\left(i\right)}^{2}+2\alpha \beta x_{\left(i\right)}^{2}+\beta^{2}x_{\left(i\right)}\right]e^{-\theta x_{\left(i\right)}}=0,\\ \frac{\partial C\left(\theta ,\alpha ,\beta \right)}{\partial \alpha }=\overset{n}{\underset{i=1}{\sum }}\left[\left(\frac{\alpha \theta +\beta +\beta \theta x_{\left(i\right)}}{\alpha \theta +\beta }\right)e^{-\theta x_{\left(i\right)}}-\frac{2n+1-2i}{2n}\right]x_{\left(i\right)}e^{-\theta x_{\left(i\right)}}=0,\\ \frac{\partial C\left(\theta ,\alpha ,\beta \right)}{\partial \beta }=\overset{n}{\underset{i=1}{\sum }}\left[\left(\frac{\alpha \theta +\beta +\beta \theta x_{\left(i\right)}}{\alpha \theta +\beta }\right)e^{-\theta x_{\left(i\right)}}-\frac{2n+1-2i}{2n}\right]x_{\left(i\right)}e^{-\theta x_{\left(i\right)}}=0. \end{array}$$

## 3. Results and Discussion

### 3.1. Simulation

To compare the five estimation methods, data were generated from the three-parameter Lindley distribution on the basis of the quantile function defined in equation (10). Data were generated for four different cases, as shown in Table 1. For each case, different sizes of samples were used (10, 30, 60, 80, 150, and 250). The experiment was repeated 10,000 times for each of combinations. Then, the parameters were estimated by the five estimation methods; the methods were compared using mean square error (MSE) and mean absolute error (MAE).  Table 2 shows the formulas of these criteria. All operations were conducted in MATLAB 2020a (see Code 1).

Tables 3–6 illustrate our simulation study. The different methods were compared based on their ranks. These results show that all estimators have the property of consistency and for all methods because MSEs and the MAEs for them decrease with an increasing sample size.

The preference of the methods can be summarised in Table 7, which shows that MPS and WLS are best for small sample sizes (10, 30). MPS, MLE, and WLS are best in medium sample sizes (60, 80), and MPS and MLE are best for large sample sizes (150, 250).

### 3.2. Application

The survival time to death for 83 COVID-19 patients was recorded by the researchers from the medical sector in Iraq/Al Anbar Province.  Table 8 contains these data.

The parameters of the three-parameter Lindley distribution were estimated by the five methods. Furthermore, the Kolmogorov-Smirnov (KS) values, $\text{KS}=\max\left|\hat{F}\left(x_{\left(i\right)}\right)-\left(i/\left(n+1\right)\right)\right|$ and their associated *p* values were calculated to ensure that these data follow the three-parameter Lindley distribution.  Table 9 shows that the data were distributed as the three-parameter Lindley distribution for all methods.

We note that all *p* values are greater than 0.05, indicating that the data follow the three-parameter Lindley distribution.

We draw p.d.f. and c.d.f. of the three-parameter Lindley distribution based on the following:

(29) $$\begin{array}{c} \hat{f}\left(t\right)=\frac{{\hat{\theta }}^{2}}{\hat{\alpha }\hat{\theta }+\hat{\beta }}\left(\hat{\alpha }+\hat{\beta }t\right)e^{-\hat{\theta }t}, \end{array}$$

(30) $$\begin{array}{c} \hat{F}\left(t\right)=1-\left[\frac{\hat{\alpha }\hat{\theta }+\hat{\beta }+\hat{\beta }\hat{\theta }t}{\hat{\alpha }\hat{\theta }+\hat{\beta }}\right]e^{-\hat{\theta }t}, \end{array}$$

where $\hat{\theta },\hat{\alpha },$ and $\hat{\beta }$ are the parameter estimates.

According to equations (29) and (30), the p.d.f. and c.d.f. can be drawn in Figures 3 and 4.

We note that the behaviour of the estimated functions is relatively close to that of the empirical functions. This finding is a good indication that the estimated models can represent the COVID-19 data.

## 4. Conclusions

The parameters of the three-parameter Lindley distribution (THPLD) were estimated by five different methods. A simulation study was performed, and these methods were compared using MSE and MAE. All estimators were consistent because their MSE and MAE values decrease as the sample size increases. The MPS and WLS methods were good in small samples. MPS, MLE, and WLS were good in medium samples. MLE and MPS were good in large samples.

On the practical side, the results indicated that the COVID-19 data follow the three-parameter Lindley distribution. The p.d.f. and c.d.f. were estimated based on the five methods, and then, these functions were drawn. The graphics indicated that the behaviour of the estimated functions is close to the empirical functions.

## Figures and Tables

**Figure 1:** The p.d.f. of the THPL distribution.

**Figure 2:** The c.d.f. of the THPL distribution.

**Figure 3:** The p.d.f. of the COVID-19 real data.

**Figure 4:** The c.d.f. of the COVID-19 real data.

**Code 1:** 

**Table 1:** Simulation cases.

Cases	*θ*	*α*	*β*
Case 1	0.25	1	2
Case 2	0.50	2	2
Case 3	0.75	2	1
Case 4	1.00	3	2

**Table 2:** Formulas of criteria.

Criteria	*θ*	*α*	*β*
MSE	$1/10000\overset{10000}{\underset{j=1}{\sum }}{\left({\hat{\theta }}_{j}-\theta \right)}^{2}$	$1/10000\overset{10000}{\underset{j=1}{\sum }}{\left({\hat{\alpha }}_{j}-\alpha \right)}^{2}$	$1/10000\overset{10000}{\underset{j=1}{\sum }}{\left({\hat{\beta }}_{j}-\beta \right)}^{2}$
MAE	$1/10000\overset{10000}{\underset{j=1}{\sum }}\left|{\hat{\theta }}_{j}-\theta \right|$	$1/10000\overset{10000}{\underset{j=1}{\sum }}\left|{\hat{\alpha }}_{j}-\alpha \right|$	$1/10000\overset{10000}{\underset{j=1}{\sum }}\left|{\hat{\beta }}_{j}-\beta \right|$

**Table 3:** Simulated MSE and MAE values for *θ* = 0.25; *α* = 1; *β* = 2.

		Methods	MLE	OLS	WLS	MPS	CVM
*n* = 10	*θ*	MSE	0.03218 ^5^	0.01026 ^4^	0.00936 ^2^	0.00842 ^1^	0.00975 ^3^
		MAE	0.11189 ^5^	0.08125 ^4^	0.07848 ^2^	0.07889 ^3^	0.07239 ^1^
	*α*	MSE	43.48015 ^5^	9.94038 ^3^	8.18130 ^2^	7.77936 ^1^	25.34155 ^4^
		MAE	9.43405 ^5^	2.61525 ^4^	2.44286 ^1^	2.47058 ^2^	2.47723 ^3^
	*β*	MSE	10.72974 ^5^	2.49457 ^3^	2.05992 ^2^	1.97869 ^1^	6.29526 ^4^
		MAE	4.68650 ^5^	1.31081 ^4^	1.22573 ^1^	1.24508 ^3^	1.24026 ^2^
		∑ ranks	30 ^5^	22 ^4^	10 ^1^	11 ^2^	17 ^3^

*n* = 30	*θ*	MSE	0.01052 ^5^	0.00310 ^3.5^	0.00244 ^1^	0.00310 ^3.5^	0.00290 ^2^
		MAE	0.05887 ^5^	0.04436 ^4^	0.03963 ^1^	0.04428 ^3^	0.04269 ^2^
	*α*	MSE	36.36728 ^5^	4.71702 ^3^	3.42387 ^1^	3.61839 ^2^	5.22673 ^4^
		MAE	2.87324 ^5^	1.73845 ^3^	1.49404 ^1^	1.52942 ^2^	1.75141 ^4^
	*β*	MSE	9.04372 ^5^	1.18165 ^3^	0.85840 ^1^	0.91062 ^2^	1.30726 ^4^
		MAE	1.43513 ^5^	0.87019 ^3^	0.74798 ^1^	0.76688 ^2^	0.87624 ^4^
		∑ ranks	30 ^5^	19.5 ^3^	6 ^1^	14.5 ^2^	20 ^4^

*n* = 60	*θ*	MSE	0.00245 ^5^	0.00118 ^4^	0.00096 ^1^	0.00116 ^3^	0.00114 ^2^
		MAE	0.02915 ^5^	0.02737 ^4^	0.02470 ^1^	0.02668 ^2^	0.02674 ^3^
	*α*	MSE	9.28063 ^5^	2.42122 ^3^	1.72204 ^2^	1.66567 ^1^	2.58512 ^4^
		MAE	1.41097 ^5^	1.21784 ^3^	1.04733 ^2^	0.99332 ^1^	1.22350 ^4^
	*β*	MSE	2.30848 ^5^	0.60595 ^3^	0.43126 ^2^	0.41808 ^1^	0.64633 ^4^
		MAE	0.70512 ^5^	0.60931 ^3^	0.52404 ^2^	0.49746 ^1^	0.61194 ^4^
		∑ ranks	30 ^5^	20 ^3^	10 ^2^	9 ^1^	21 ^4^

*n* = 80	*θ*	MSE	0.00245 ^5^	0.00118 ^4^	0.00096 ^1^	0.00116 ^3^	0.00114 ^2^
		MAE	0.02915 ^5^	0.02737 ^4^	0.02470 ^1^	0.02668 ^2^	0.02674 ^3^
	*α*	MSE	9.28063 ^5^	2.42122 ^3^	1.72204 ^2^	1.66567 ^1^	2.58512 ^4^
		MAE	1.41097 ^5^	1.21784 ^3^	1.04733 ^2^	0.99332 ^1^	1.22350 ^4^
	*β*	MSE	2.30848 ^5^	0.60595 ^3^	0.43126 ^2^	0.41808 ^1^	0.64633 ^4^
		MAE	0.70512 ^5^	0.60931 ^3^	0.52404 ^2^	0.49746 ^1^	0.61194 ^4^
		∑ ranks	30 ^5^	20 ^3^	10 ^2^	9 ^1^	21 ^4^

*n* = 150	*θ*	MSE	0.00039 ^2^	0.00053 ^4^	0.00042 ^3^	0.00038 ^1^	0.00054 ^5^
		MAE	0.01570 ^2^	0.01836 ^4^	0.01654 ^3^	0.01553 ^1^	0.01860 ^5^
	*α*	MSE	0.64435 ^2^	0.93673 ^4^	0.68549 ^3^	0.57175 ^1^	0.97507 ^5^
		MAE	0.61355 ^2^	0.76963 ^4^	0.66373 ^3^	0.57905 ^1^	0.78293 ^5^
	*β*	MSE	0.16115 ^2^	0.23441 ^4^	0.17157 ^3^	0.14333 ^1^	0.24391 ^5^
		MAE	0.30685 ^2^	0.38495 ^4^	0.33199 ^3^	0.28980 ^1^	0.39155 ^5^
		∑ ranks	12 ^2^	24 ^4^	18 ^3^	6 ^1^	30 ^5^

*n* = 250	*θ*	MSE	0.00021 ^1^	0.00030 ^4.5^	0.00024 ^3^	0.00022 ^2^	0.00030 ^4.5^
		MAE	0.01153 ^1^	0.01358 ^4.5^	0.01211 ^3^	0.01178 ^2^	0.01358 ^4.5^
	*α*	MSE	0.34852 ^2^	0.57886 ^4^	0.40969 ^3^	0.32996 ^1^	0.58881 ^5^
		MAE	0.46014 ^2^	0.59850 ^4^	0.51026 ^3^	0.45677 ^1^	0.60467 ^5^
	*β*	MSE	0.08713 ^2^	0.14483 ^4^	0.10250 ^3^	0.08265 ^1^	0.14728 ^5^
		MAE	0.23008 ^2^	0.29933 ^4^	0.25519 ^3^	0.22853 ^1^	0.30239 ^5^
		∑ ranks	10 ^2^	25 ^4^	18 ^3^	8 ^1^	29 ^5^

**Table 4:** Simulated MSE and MAE values for *θ* = 0.5; *α* = 2; *β* = 2.

		Methods	MLE	OLS	WLS	MPS	CVM
*n* = 10	*θ*	MSE	0.14601 ^5^	0.03947 ^3^	0.03631 ^1^	0.03684 ^2^	0.05132 ^4^
		MAE	0.23835 ^5^	0.16298 ^2^	0.15646 ^1^	0.16313 ^3^	0.16916 ^4^
	*α*	MSE	71.23759 ^5^	3.82925 ^1^	4.12533 ^2^	5.03375 ^3^	17.29708 ^4^
		MAE	4.17613 ^5^	1.58224 ^3^	1.48048 ^2^	1.41634 ^1^	1.92063 ^4^
	*β*	MSE	67.78865 ^5^	3.79938 ^1^	4.08219 ^2^	5.00455^3^	16.18706 ^4^
		MAE	4.07386 ^5^	1.58602 ^3^	1.48560 ^2^	1.43176 ^1^	1.91369 ^4^
		∑ ranks	30 ^5^	13 ^2.5^	10 ^1^	13 ^2.5^	24 ^4^

*n* = 30	*θ*	MSE	0.02479 ^5^	0.01491 ^2^	0.01405 ^1^	0.01557 ^4^	0.01536 ^3^
		MAE	0.10212 ^5^	0.09886 ^3^	0.09431 ^1^	0.10131 ^4^	0.09720 ^2^
	*α*	MSE	3.76396 ^5^	1.84640 ^3^	1.65069 ^2^	1.55848 ^1^	2.15370 ^4^
		MAE	1.28676 ^5^	1.11793 ^3^	1.06370 ^2^	1.03561 ^1^	1.17191 ^4^
	*β*	MSE	3.76245 ^5^	1.84675 ^3^	1.65356 ^2^	1.57176 ^1^	2.15014 ^4^
		MAE	1.28701 ^5^	1.11841 ^3^	1.06473 ^2^	1.03957 ^1^	1.17156 ^4^
		∑ ranks	30 ^5^	17 ^3^	10 ^1^	12 ^2^	21 ^4^

*n* = 60	*θ*	MSE	0.00749 ^1^	0.00977 ^5^	0.00786 ^2^	0.00959 ^4^	0.00931 ^3^
		MAE	0.06596 ^1^	0.07759 ^5^	0.07002 ^2^	0.07591 ^4^	0.07478 ^3^
	*α*	MSE	1.20820 ^4^	1.19844 ^3^	1.02540 ^1^	1.04832 ^2^	1.25362 ^5^
		MAE	0.84381 ^3^	0.90047 ^4^	0.82780 ^2^	0.82641 ^1^	0.90760 ^5^
	*β*	MSE	1.20128 ^4^	1.19806 ^3^	1.02577 ^1^	1.05479 ^2^	1.25156 ^5^
		MAE	0.84338 ^3^	0.90057 ^4^	0.82819 ^1^	0.82857 ^2^	0.90729 ^5^
		∑ ranks	16 ^3^	24 ^4^	9 ^1^	15 ^2^	26 ^5^

*n* = 80	*θ*	MSE	0.00488 ^1^	0.00701 ^5^	0.00579 ^2^	0.00681 ^4^	0.00664 ^3^
		MAE	0.05512 ^1^	0.06602 ^5^	0.06049 ^2^	0.06323 ^3^	0.06381 ^4^
	*α*	MSE	0.75079 ^1^	0.95293 ^4^	0.80563 ^3^	0.80042 ^2^	0.97670 ^5^
		MAE	0.70061 ^1^	0.78612 ^4^	0.72550 ^3^	0.71594 ^2^	0.78956 ^5^
	*β*	MSE	0.75088 ^1^	0.95296 ^4^	0.80621 ^3^	0.80450 ^2^	0.97609 ^5^
		MAE	0.70075 ^1^	0.78637 ^4^	0.72589 ^3^	0.71736 ^2^	0.78963 ^5^
		∑ ranks	6 ^1^	26 ^4^	16 ^3^	15 ^2^	27 ^5^

*n* = 150	*θ*	MSE	0.00249 ^1^	0.00332 ^5^	0.00275 ^2^	0.00321 ^4^	0.00318 ^3^
		MAE	0.03992 ^1^	0.04539 ^5^	0.04172 ^2^	0.04429 ^3^	0.04483 ^4^
	*α*	MSE	0.43720 ^1^	0.51020 ^4^	0.44399 ^2^	0.47251 ^3^	0.51644 ^5^
		MAE	0.53520 ^1^	0.58229 ^5^	0.54531 ^2^	0.56199 ^3^	0.58181 ^4^
	*β*	MSE	0.43716 ^1^	0.51061 ^4^	0.44431 ^2^	0.47378 ^3^	0.51656 ^5^
		MAE	0.53527 ^1^	0.58256 ^5^	0.54552 ^2^	0.56257 ^3^	0.58196 ^4^
		∑ ranks	6 ^1^	28 ^5^	12 ^2^	19 ^3^	25 ^4^

*n* = 250	*θ*	MSE	0.00141 ^1^	0.00192 ^5^	0.00158 ^2^	0.00164 ^3^	0.00189 ^4^
		MAE	0.02956 ^1^	0.03486 ^5^	0.03149 ^3^	0.03131 ^2^	0.03472 ^4^
	*α*	MSE	0.24155 ^1^	0.31334 ^4^	0.26297 ^3^	0.25504 ^2^	0.31684 ^5^
		MAE	0.38629 ^1^	0.44107 ^4^	0.40250 ^3^	0.39923 ^2^	0.44152 ^5^
	*β*	MSE	0.24191 ^1^	0.31359 ^4^	0.26327 ^3^	0.25568 ^2^	0.31696 ^5^
		MAE	0.38651 ^1^	0.44125 ^4^	0.40268 ^3^	0.39960 ^2^	0.44163 ^5^
		∑ ranks	6 ^1^	26 ^4^	17 ^3^	13 ^2^	28 ^5^

**Table 5:** Simulated MSE and MAE values for *θ* = 0.75; *α* = 2; *β* = 1.

		Methods	MLE	OLS	WLS	MPS	CVM
*n* = 10	*θ*	MSE	0.46095 ^5^	0.10901 ^3^	0.10492 ^2^	0.09316 ^1^	0.20454 ^4^
		MAE	0.40706 ^5^	0.25315 ^3^	0.25002 ^2^	0.24814 ^1^	0.32268 ^4^
	*α*	MSE	7.30773 ^5^	0.88762 ^3^	0.75417 ^2^	0.36515 ^1^	1.97648 ^4^
		MAE	1.28431 ^5^	0.68135 ^3^	0.65473 ^2^	0.50256 ^1^	1.02787 ^4^
	*β*	MSE	24.59881 ^5^	3.39581 ^3^	2.90920 ^2^	1.43334 ^1^	7.55938 ^4^
		MAE	2.35659 ^5^	1.35906 ^3^	1.30658 ^2^	1.00570 ^1^	2.04089 ^4^
		∑ ranks	30 ^5^	18 ^3^	12 ^2^	6 ^1^	24 ^4^

*n* = 30	*θ*	MSE	0.06690 ^5^	0.04853 ^3^	0.04496 ^2^	0.04316 ^1^	0.05869 ^4^
		MAE	0.18291 ^4^	0.17765 ^3^	0.17162 ^1^	0.17480 ^2^	0.18997 ^5^
	*α*	MSE	1.58905 ^5^	0.46849 ^3^	0.44001 ^2^	0.28803 ^1^	0.67987 ^4^
		MAE	0.63403 ^5^	0.53905 ^3^	0.52523 ^2^	0.44839 ^1^	0.63214 ^4^
	*β*	MSE	5.98867 ^5^	1.82556 ^3^	1.71402 ^2^	1.12452 ^1^	2.63263 ^4^
		MAE	1.26566 ^5^	1.07315 ^3^	1.04227 ^2^	0.89183 ^1^	1.25457 ^4^
		∑ ranks	29 ^5^	18 ^3^	11 ^2^	7 ^1^	25 ^4^

*n* = 60	*θ*	MSE	0.02559 ^1^	0.03494 ^4^	0.03086 ^3^	0.02900 ^2^	0.03860 ^5^
		MAE	0.13036 ^1^	0.15528 ^4^	0.14667 ^3^	0.14479 ^2^	0.15984 ^5^
	*α*	MSE	0.33048 ^4^	0.32315 ^3^	0.31141 ^2^	0.22678 ^1^	0.40365 ^5^
		MAE	0.44401 ^2^	0.46366 ^4^	0.45053 ^3^	0.40967 ^1^	0.50794 ^5^
	*β*	MSE	1.30500 ^4^	1.27351 ^3^	1.20807 ^2^	0.89143 ^1^	1.58622 ^5^
		MAE	0.88645 ^2^	0.92364 ^4^	0.89209 ^3^	0.81442 ^1^	1.01055 ^5^
		∑ ranks	14 ^2^	22 ^4^	16 ^3^	8 ^1^	30 ^5^

*n* = 80	*θ*	MSE	0.01956 ^1^	0.02630 ^4^	0.02362 ^2^	0.02502 ^3^	0.02632 ^5^
		MAE	0.11415 ^1^	0.13715 ^5^	0.12847 ^2^	0.13238 ^3^	0.13510 ^4^
	*α*	MSE	0.22090 ^3^	0.22234 ^4^	0.21826 ^2^	0.18003 ^1^	0.25653 ^5^
		MAE	0.37883 ^2^	0.39558 ^4^	0.39210 ^3^	0.36513 ^1^	0.41496 ^5^
	*β*	MSE	0.87142 ^3^	0.87899 ^4^	0.85417 ^2^	0.70862 ^1^	1.01140 ^5^
		MAE	0.75581 ^2^	0.78851 ^4^	0.77820 ^3^	0.72630 ^1^	0.82649 ^5^
		∑ ranks	12 ^2^	25 ^4^	14 ^3^	10 ^1^	29 ^5^

*n* = 150	*θ*	MSE	0.01352 ^1^	0.01917 ^5^	0.01562 ^2^	0.01717 ^3^	0.01851 ^4^
		MAE	0.09182 ^1^	0.11387 ^5^	0.10079 ^2^	0.10565 ^3^	0.11101 ^4^
	*α*	MSE	0.13580 ^2^	0.15468 ^4^	0.14046 ^3^	0.12917 ^1^	0.16394 ^5^
		MAE	0.28566 ^1^	0.32341 ^4^	0.29892 ^3^	0.29498 ^2^	0.32868 ^5^
	*β*	MSE	0.53845^2^	0.61391 ^4^	0.55081 ^3^	0.50980^1^	0.65031 ^5^
		MAE	0.57037 ^1^	0.64527 ^4^	0.59372 ^3^	0.58739 ^2^	0.65573 ^5^
		∑ ranks	8 ^1^	26 ^4^	16 ^3^	12 ^2^	28 ^5^

*n* = 250	*θ*	MSE	0.00853 ^1^	0.01271^5^	0.01014 ^2^	0.01232 ^4^	0.01221 ^3^
		MAE	0.07247 ^1^	0.08780 ^4^	0.07840 ^2^	0.08488 ^3^	0.08678 ^5^
	*α*	MSE	0.08640 ^1^	0.10876 ^4^	0.09533 ^3^	0.09198 ^2^	0.11249 ^5^
		MAE	0.23346 ^1^	0.26235 ^4^	0.24618 ^3^	0.24553 ^2^	0.26498 ^5^
	*β*	MSE	0.34281 ^1^	0.43149 ^4^	0.37524 ^3^	0.36396 ^2^	0.44615 ^5^
		MAE	0.46586 ^1^	0.52343 ^4^	0.48985 ^3^	0.48908 ^2^	0.52865 ^5^
		∑ ranks	6 ^1^	25 ^4^	16 ^3^	15 ^2^	28 ^5^

**Table 6:** Simulated MSE and MAE values for *θ* = 1; *α* = 3; *β* = 2.

		Methods	MLE	OLS	WLS	MPS	CVM
*n* = 10	*θ*	MSE	0.70679 ^5^	0.20333 ^3^	0.18211 ^2^	0.14954 ^1^	0.34231 ^4^
		MAE	0.49513 ^5^	0.32538 ^3^	0.30905 ^2^	0.30597 ^1^	0.39874 ^4^
	*α*	MSE	9.65813 ^5^	2.57452 ^3^	2.27693 ^2^	1.78596 ^1^	4.33115 ^4^
		MAE	2.02567 ^5^	1.39712 ^3^	1.31386 ^2^	1.18546 ^1^	1.75046 ^4^
	*β*	MSE	23.59916 ^5^	5.91723 ^3^	5.29318 ^2^	4.13198 ^1^	9.98005 ^4^
		MAE	3.12830 ^5^	2.11840 ^3^	2.00008 ^2^	1.80460 ^1^	2.65809 ^4^
		∑ ranks	30 ^5^	18 ^3^	12 ^2^	6 ^1^	24 ^4^

*n* = 30	*θ*	MSE	0.11144 ^4^	0.10159 ^3^	0.09699 ^2^	0.08264 ^1^	0.12154 ^5^
		MAE	0.24409 ^1^	0.25875 ^4^	0.25245 ^3^	0.24785 ^2^	0.27211 ^5^
	*α*	MSE	2.11424 ^4^	2.04946 ^3^	1.98698 ^2^	1.49819 ^1^	2.44848 ^5^
		MAE	1.19660 ^2^	1.24289 ^4^	1.22727 ^3^	1.10448 ^1^	1.32051 ^5^
	*β*	MSE	4.81637 ^4^	4.65230 ^3^	4.52961 ^2^	3.42073 ^1^	5.55365 ^5^
		MAE	1.80455 ^2^	1.87439 ^4^	1.85195 ^3^	1.67023 ^1^	1.99037 ^5^
		∑ ranks	17 ^3^	21 ^4^	15 ^2^	7 ^1^	30 ^5^

*n* = 60	*θ*	MSE	0.04638 ^1^	0.05668 ^4^	0.05298 ^2^	0.05632 ^3^	0.05752 ^5^
		MAE	0.17603 ^1^	0.20285 ^4^	0.19396 ^2^	0.20489 ^5^	0.19851 ^3^
	*α*	MSE	1.18298 ^2^	1.29965 ^4^	1.22888 ^3^	1.12028 ^1^	1.40697 ^5^
		MAE	0.90122 ^1^	0.98171 ^4^	0.94750 ^3^	0.91717 ^2^	1.00321 ^5^
	*β*	MSE	2.64623 ^2^	2.94626 ^4^	2.77000 ^3^	2.54612 ^1^	3.18810 ^5^
		MAE	1.35253 ^1^	1.47795 ^4^	1.42273 ^3^	1.38288 ^2^	1.51001 ^5^
		∑ ranks	8 ^1^	24 ^4^	16 ^3^	14 ^2^	28 ^5^

*n* = 80	*θ*	MSE	0.03774 ^1^	0.04979 ^4^	0.04402 ^2^	0.04442 ^3^	0.05140 ^5^
		MAE	0.15914 ^1^	0.18567 ^4^	0.17370 ^2^	0.17625 ^3^	0.18767 ^5^
	*α*	MSE	0.99836 ^2^	1.13319 ^4^	1.06474 ^3^	0.96882 ^1^	1.21750 ^5^
		MAE	0.82878 ^1^	0.90220 ^4^	0.87451 ^3^	0.85537 ^2^	0.92640 ^5^
	*β*	MSE	2.25457 ^2^	2.56297 ^4^	2.39748 ^3^	2.20537 ^1^	2.75261 ^5^
		MAE	1.24645 ^1^	1.35657 ^4^	1.31250 ^3^	1.28998 ^2^	1.39279 ^5^
		∑ ranks	8 ^1^	24 ^4^	16 ^3^	12 ^2^	30 ^5^

*n* = 150	*θ*	MSE	0.02392 ^1^	0.03347 ^5^	0.02822 ^2^	0.03321 ^4^	0.03228 ^3^
		MAE	0.12421 ^1^	0.14950 ^5^	0.13665 ^2^	0.14758 ^4^	0.14688 ^3^
	*α*	MSE	0.61928 ^1^	0.75490 ^4^	0.67782 ^2^	0.72412 ^3^	0.75762 ^5^
		MAE	0.64467 ^1^	0.73119 ^5^	0.68630 ^2^	0.71184 ^3^	0.72699 ^4^
	*β*	MSE	1.39973 ^1^	1.70290 ^4^	1.52836 ^2^	1.64596 ^3^	1.70962 ^5^
		MAE	0.96927 ^1^	1.09756 ^5^	1.03002 ^2^	1.07266 ^3^	1.09141 ^4^
		∑ ranks	6 ^1^	28 ^5^	12 ^2^	20 ^3^	24 ^4^

*n* = 250	*θ*	MSE	0.01411 ^1^	0.02180 ^5^	0.01702 ^2^	0.01995 ^3^	0.02099 ^4^
		MAE	0.09269 ^1^	0.11508 ^5^	0.10070 ^2^	0.10868 ^3^	0.11370 ^4^
	*α*	MSE	0.40840 ^1^	0.55654 ^5^	0.46808 ^2^	0.49339 ^3^	0.55312 ^4^
		MAE	0.50869 ^1^	0.60068 ^5^	0.54687 ^2^	0.56429 ^3^	0.59688 ^4^
	*β*	MSE	0.92151 ^1^	1.25077 ^5^	1.05215 ^2^	1.12009 ^3^	1.24249 ^4^
		MAE	0.76418 ^1^	0.90062 ^5^	0.81990 ^2^	0.84957 ^3^	0.89478 ^4^
		∑ ranks	6 ^1^	30 ^5^	12 ^2^	18 ^3^	24 ^4^

**Table 7:** Best methods based on the simulation study.

Cases	*n* = 10	*n* = 30	*n* = 60	*n* = 80	*n* = 150	*n* = 250
Case 1	WLS	WLS	MPS	MPS	MPS	MPS
Case 2	WLS	WLS	WLS	MLE	MLE	MLE
Case 3	MPS	MPS	MPS	MPS	MLE	MLE
Case 4	MPS	MPS	MLE	MLE	MLE	MLE

**Table 8:** Survival time for 83 patients (in days).

1	1	1	1	1	1	1	1	2	2	2	2	2	2	2	2	2	3
3	3	3	3	3	3	4	4	4	4	4	4	4	5	5	5	5	5
6	6	6	6	6	7	7	7	7	7	7	8	8	8	8	8	9	9
9	10	10	10	10	10	10	10	11	11	11	12	12	12	12	12	12	13
13	13	18	19	20	20	21	22	22	22	23							

**Table 9:** Parameter estimates under all methods, K-S statistics, and the associated *p* values for the COVID-19 data.

Methods	$\hat{\theta }$	$\hat{\alpha }$	$\hat{\beta }$	KS	*p* values
MLE	0.2493	1.4578	4.3020	0.0890	0.4982
OLS	0.2186	3.1600	1.7605	0.0583	0.9248
WLS	0.2363	2.4292	2.8594	0.0711	0.7684
MPS	0.2350	2.4132	2.8762	0.0727	0.7445
CVM	0.2236	3.0096	1.9856	0.0554	0.9485

## Data Availability

Data are available upon request from the authors.
